# The Effects of Statin Therapy on Oxidized LDL and Its Antibodies: A Systematic Review and Meta-Analysis

**DOI:** 10.1155/2022/7850659

**Published:** 2022-08-01

**Authors:** Tannaz Jamialahmadi, Fatemeh Baratzadeh, Željko Reiner, Massimo R. Mannarino, Vladimiro Cardenia, Luis E. Simental-Mendía, Matteo Pirro, Gerald F. Watts, Amirhossein Sahebkar

**Affiliations:** ^1^Surgical Oncology Research Center, Mashhad University of Medical Sciences, Mashhad, Iran; ^2^Department of Clinical Pharmacy, School of Pharmacy, Isfahan University of Medical Sciences, Isfahan, Iran; ^3^Department of Internal Medicine, University Hospital Centre Zagreb, School of Medicine, University of Zagreb, Zagreb, Croatia; ^4^Unit of Internal Medicine, Angiology and Arteriosclerosis Diseases, Department of Medicine, University of Perugia, Perugia, Italy; ^5^Department of Agricultural, Forest and Food Sciences (DISAFA), University of Turin, Grugliasco 10095, Italy; ^6^Biomedical Research Unit, Mexican Social Security Institute, Durango, Mexico; ^7^Cardiometabolic Service, Department of Cardiology, Royal Perth Hospital, School of Medicine, The University of Western Australia, Perth, Western Australia, Australia; ^8^Applied Biomedical Research Center, Mashhad University of Medical Sciences, Mashhad, Iran; ^9^Biotechnology Research Center, Pharmaceutical Technology Institute, Mashhad University of Medical Sciences, Mashhad, Iran; ^10^Department of Biotechnology, School of Pharmacy, Mashhad University of Medical Sciences, Mashhad, Iran

## Abstract

**Background:**

Elevated serum low-density lipoproteins (LDL), the substrate for the formation of atherogenic oxidized LDLs (oxLDL), are a causal factor for atherosclerotic cardiovascular disease (ASCVD). Statins are well known to decrease LDL particle concentration and reduce ASCVD morbidity and mortality.

**Objective:**

To perform a meta-analysis of the effects of statins (i.e., type, dose, and duration of treatment) on serum levels of oxLDL and on immunoglobulin M (IgM) and immunoglobulin G (IgG) antibody levels against oxLDL.

**Methods:**

PubMed, Scopus, Embase, and Web of Science were searched up to February 5th, 2021, for randomized controlled trials (RCT) evaluating the effect of statins on oxLDL and anti-oxLDL antibody levels. Meta-analysis was performed using Comprehensive Meta-Analysis (CMA) V2 software. To evaluate the influence of each study on the overall effect size, a sensitivity analysis was performed using the leave-one-out method. Evaluation of the funnel plot, Begg's rank correlation, and Egger's weighted regression tests was used to assess the presence of publication bias in the meta-analysis.

**Results:**

A total of 28 RCTs including 4019 subjects were finally included in the meta-analysis. The results indicated a significant decrease in circulating concentrations of oxLDL after treatment with statins (SMD: -2.150, 95% CI: -2.640, -1.697, *p* < 0.001). Subgroup analysis found no significant effect of the intensity of statin treatment or statin lipophilicity on the reduction of circulating concentrations of oxLDL. An additional meta-analysis of 3 trials showed that statins did not change the serum levels of IgM and IgG antibodies to oxLDL.

**Conclusion:**

Statin therapy decreases serum oxLDL concentrations but does not affect circulating levels of anti-oxLDL antibodies.

## 1. Introduction

Elevated serum low-density lipoprotein cholesterol (LDL-C) is a causal factor for atherosclerotic cardiovascular disease (ASCVD) morbidity and mortality [1]. Statins are drugs of choice to decrease LDL-C levels and ASCVD risk in both primary and secondary prevention [2, 3]. The oxidation of LDL particles, which typically occurs in patients with elevated LDL-C levels as well as in the presence of other prooxidative conditions, is considered to be the major atherogenic modification of LDL [4]. Among LDL subclasses, small and very small dense particles are most susceptible to oxidation [5]. Oxidized LDL (oxLDL) can trigger the expression of adhesion molecules (e.g., intracellular adhesion molecule-1 (ICAM-1), vascular adhesion molecule-1 (VCAM-1), and E-selectin) on the endothelial cell surface resulting in activation of endothelial cells [6, 7]. These adhesion molecules along with integrins, selectins, and chemokines stimulate the recruitment and adhesion of leukocytes, mostly monocytes, to the endothelium and their infiltration into intima. Monocytes differentiate to macrophages, recognize and internalize oxLDL particles by scavenger receptors, and transform into foam cells, thus initiating the formation of the atherosclerotic plaque [8]. Moreover, the overexpression of the lectin-like oxidized low-density lipoprotein receptor-1 (LOX-1), the main oxLDL receptor in endothelial cells, promotes endothelial cell activation and dysfunction, triggering the activation of proinflammatory signaling pathways and the development of atherosclerotic process [9]. oxLDL particles participate in the destabilization of atherosclerotic plaques leading to clinical manifestations, such as myocardial infarction (MI) and unstable angina. In addition to promoting plaque appearance, growth, inflammation, and destabilization, oxLDLs act as immune antigens inducing the innate immune response to produce immunoglobulin M (IgM) and immunoglobulin G (IgG) antibodies against oxLDL [8]. The role of these antibodies as markers of oxLDL exposure and pathogenic determinants of ASCVD has been proposed [10]. Namely, as a consequence of the macrophage activation, matrix metalloproteinases are produced causing matrix degradation, fissuring of the plaque, and thrombus formation on this site [11].

In the armamentarium of different lipid-lowering drugs [12–14], statins still remain the most widely prescribed class. This is due to their efficient LDL-lowering activity and pleiotropic effects of these drugs ([15–21]). Although the effects of statins on LDL-C are well known, inconsistency about the effects of statin therapy on circulating levels of oxLDL and anti-oxLDL antibodies is still present. Moreover, the impact of statin therapy intensity and lipophilicity on these highly atherogenic modified LDL particles remains unexplored, and it is not known whether different statins have different effects on serum concentrations of oxLDL. Therefore, the aim of this systematic review and meta-analysis was to analyze the magnitude of the effect of statins on oxLDL and anti-oxLDL antibody levels.

## 2. Methods

### 2.1. Search Strategy

We followed the methods of Jamialahmadi et al. as follows [22]. The present systematic review and meta-analysis was designed according to the 2009 Preferred Reporting Items for Systematic Reviews and Meta-Analysis (PRISMA) guidelines [23]. PubMed, Scopus, Embase, and Web of Science were searched from inception to February 5th, 2021, using the following keywords in titles and abstracts (also in combination with MESH terms): (“Hydroxymethylglutaryl-CoA Reductase Inhibitors” OR simvastatin OR rosuvastatin OR atorvastatin OR pravastatin OR pitavastatin OR mevastatin OR fluvastatin OR lovastatin OR cerivastatin) AND (“oxidized low density lipoprotein” OR “oxidized LDL” OR OxLDL OR ox-LDL OR “oxidized Low-Density Lipoprotein” OR “minimally modified oxidized-LDL” OR MM-LDL OR MMLDL OR “malondialdehyde-low density lipoprotein” OR “malondialdehyde low density lipoprotein” OR “MDA-LDL” OR “MDALDL” OR “MDA-LDL IgM” OR “MDA-LDL IgG” OR “autoantibodies against oxidized low-density lipoprotein” OR “autoantibodies against oxidized low density lipoprotein” OR “AuAb-oxLDL” OR “antibodies against oxidized LDL” OR “Anti-oxLDL”). The search was performed consecutively using the search engines and search terms which are presented in Supplementary Material Table S1.

### 2.2. Study Selection

Human studies were included if they met the following inclusion criteria: (i) randomized controlled trial with either parallel or cross-over design, (ii) the study which investigated the effect of statins on oxLDL and/or antibodies against oxLDL, and (iii) presentation of sufficient information at baseline and at the end of follow-up in each group or studies which provided the net change values. Exclusion criteria were as follows: (i) nonrandomized trials, (ii) uncontrolled trials, (iii) observational studies with case-control, cross-sectional, or cohort design, and (iv) lack of sufficient information at baseline or follow-up and of an active comparator in the control group.

### 2.3. Data Extraction

We followed the methods of Jamialahmadi et al. as follows [22]. After removal of duplicate studies, two independent and blinded authors (JB, MR) evaluated eligibility by screening the titles and abstracts of the studies. Full reports of eligible studies were obtained. Any disagreements were resolved by discussion and consensus. Eligible studies were reviewed, and the following data were abstracted: (1) the name of the first author, (2) the year of publication, (3) study design, (4) type of statins used in the study, (5) dose of statin, (6) treatment duration, (7) patient characteristics, and (8) clinical outcomes.

### 2.4. Quality Assessment

We followed the methods of Jamialahmadi et al. as follows [22]. Risk of bias in the studies included in this meta-analysis was evaluated according to the Cochrane instructions [24]. Selection bias, performance bias, attrition bias, detection bias, reporting bias, and other sources of bias were estimated to be high, low, or unclear for each of the included studies.

### 2.5. Quantitative Data Synthesis

We followed the methods of Jamialahmadi et al. as follows [22]. Meta-analysis was performed using Comprehensive Meta-Analysis (CMA) V2 software (Biostat, NJ) [25]. Values were reported in different units. Sample sizes, means, and standard deviations from each group were obtained for each relevant outcome to calculate standardized mean differences (SMDs). We applied SMDs because of the different metrics used to assess outcomes. Effect size was calculated as (measured at the end of follow − up in the treatment group − measured at baseline in the treatment group) − (measured at the end of follow‐up in the control group − measured at baseline in the control group). A random-effects model and the generic inverse variance weighting method were used to compensate for the heterogeneity of the studies in terms of study design, treatment duration, and the characteristics of the studied populations [23]. If the outcome measures were reported in the median and range (or 95% confidence interval (CI)), mean and SD values were estimated using the method described by Hozo et al. [26]. Where only the standard error of the mean (SEM) was reported, SD was estimated using the following formula: SD = SEM × sqrt (*n*), where *n* is the number of subjects. Given the variations in the assay methods and reporting different oxLDL concentrations, effect sizes were expressed as SMD and 95% CI. To evaluate the influence of each study on the overall effect size, a sensitivity analysis was performed using the leave-one-out method (i.e., removing one study each time and repeating the analysis) [27, 28].

### 2.6. Metaregression

We followed the methods of Jamialahmadi et al. as follows [22]. As potential confounders of treatment response, the baseline levels of oxLDL and duration of statin treatment were included into a random-effects metaregression model to explore their association with the estimated effect size.

### 2.7. Publication Bias

We followed the methods of Jamialahmadi et al. as follows [22]. Evaluation of the funnel plot, Begg's rank correlation, and Egger's weighted regression tests was used to assess the presence of publication bias in the meta-analysis. When there was evidence of funnel plot asymmetry, potentially missing studies were included using the “trim and fill” method. In case of a significant result, the number of potentially missing studies required to make the *p* value nonsignificant was estimated using the “fail-safe *N*” method as another marker of publication bias [29].

### 2.8. GRADE Scoring

We assessed the strength of evidence for each outcome using the Grading of Recommendations, Assessment, Development and Evaluation (GRADE) system [30]. GRADEpro GDT software was used to summarise the finding for each outcome, which is presented in Supplementary Material Table S2. According to the GRADE system, RCTs start as high-quality evidence. Four points were given for each outcome, and then, we assessed factors reducing the quality of the evidence. For each outcome, points were reduced based on the presence of the following: the overall risk of bias for each RCT, inconsistency, indirectness, and imprecision. Accordingly, we graded the evidence in four categories based on the overall GRADE scores for each intervention: high-grade evidence (at least 4 points), moderate-grade evidence (3 points), low-grade evidence (2 points), and very low-grade evidence (1 point).

## 3. Results

Among the 1444 published studies identified by a systematic database search, 134 were directly related to the topic of this study. However, 106 studies were excluded after careful evaluation (3 studies were cross-sectional, 21 studies were not found, 24 studies were not randomized clinical trials, 39 studies did not report sufficient data, 36 studies were actively controlled, 22 studies were poster presentations, and 1 study investigated cerivastatin, a drug currently withdrawn from almost all markets). Therefore, 28 RCTs were finally included in the systematic review and meta-analysis. A total of 25 studies evaluated the circulating concentrations of oxLDL and malondialdehyde (MDA) LDL (Table 1), while 3 studies measured antibodies against oxLDL and MDA LDL (Table 2). The study selection process is shown in Figure 1.

### 3.1. Risk of Bias Assessment of Clinical Trials

Most of the selected trials showed insufficient information regarding both random sequence generation and allocation concealment. Furthermore, seven studies showed a high risk of bias for blinding of participants, personnel, and outcome assessment [40, 46, 49, 52, 54]. Finally, all included trials had a low risk of bias for incomplete outcome data and selective reporting. The evaluation of the risk of bias in the selected studies is presented in Figure 2.

### 3.2. Assays for oxLDL

In most of the included studies, serum oxLDL was measured using the enzyme-linked immunosorbent assay (ELISA) method. Thirteen studies used the Mercodia oxLDL kit (Mercodia, Uppsala, Sweden) [31–37, 44, 45, 47–49, 55], three studies used the SRL kit (Tokyo, Japan) [39, 40, 51], one study used the USCNK Life Science Inc. kit (Wuhan, China) [41], one study used the R&D Systems Inc. kit (Minneapolis, Minnesota, USA) [42], one study used the Immundiagnostik kit (Bensheim, Germany) [43], one study used the Kyowa Medex MX kit (Kyowa Medex, Inc., Tokyo) [50], one study used the Daiichi kit (Tokyo, Japan) [52], one study used the Biomedica kit (Wien, Austria) [57], one study used ML25 (monoclonal antibody against MDA-LDL) [54], and five studies did not mention the methods used or assay kits [38, 46, 53, 56, 58].

### 3.3. Effect of Statins on Circulating Concentrations of Oxidized LDL

Meta-analysis from 25 trials including 1444 subjects demonstrated a significant decrease in circulating concentrations of oxLDL (SMD: -2.150, 95% CI: -2.604, -1.697, *p* < 0.001) (Figure 3(a)). The reduction in circulating concentrations of oxLDL because of statin treatment was robust in the leave-one-out sensitivity analysis (Figure 3(b)).

### 3.4. Effect of Statins on Antibodies to Oxidized LDL (IgG and IgM)

Meta-analysis from 3 clinical trials including 2575 subjects did not show a significant change in serum IgM antibodies to oxLDL (SMD: -10.842, 95% CI: -32.091, 10.406, *p* = 0.317) and IgG (SMD: 0.048, 95% CI: -0.030, 0.125, *p* = 0.229) following treatment with statins (Figures 4(a) and 4(b)).

### 3.5. Metaregression

Random-effects metaregression was performed to assess the effect of potential confounders on the circulating concentrations of oxLDL-lowering activity of statins. The results did not suggest any significant association between the changes in circulating concentrations of oxLDL and either baseline level (slope: -0.00069; 95% CI: -0.00685, 0.00547; *p* = 0.826), treatment duration (slope: 0.0255; 95% CI: -0.00961, 0.06068; *p* = 0.154), or delta LDL (slope: -0.0121; 95% CI: -0.0591, 0.0349; *p* = 0.613) (Figures 5(a)–5(c)).

### 3.6. Subgroup Analysis

A subgroup analysis was also performed based on statin type and lipophilicity, statin dose, and treatment duration (≤12 weeks and >12 weeks). Subgroup analyses showed significant associations between the statin type and oxLDL level changes (*p* = 0.024). There was no significant effect of statin lipophilicity (*p* = 0.102) and doses (*p* = 0.491) on the reduction of circulating concentrations of oxLDL. A negative association between the treatment duration and change in oxLDL levels (*p* = 0.039) was found (Table 3).

### 3.7. Publication Bias

Given the asymmetric funnel plot, Egger's linear regression test (intercept = −7.33, standard error = 0.83; 95%CI = −9.04, −5.62, *t* = 8.79, df = 28, two-tailed *p* < 0.001) and Begg's rank correlation test (Kendall′s tau with continuity correction = −0.48, *z* = 3.74, two-tailed *p* value < 0.001) suggest the presence of publication bias in the meta-analysis of the effects of statins on serum oxLDL and antibodies. Using the “trim and fill” method, three potentially missing studies were included showing an adjusted effect size (SMD) of -2.53 (95% CI: -3.12, -1.93). The “fail-safe *N*” test showed that 4904 missing studies would be needed to bring the effect size down to a nonsignificant (*p* > 0.05) value (Figure 6).

## 4. Discussion

The results of our meta-analysis suggest that treatment with statins significantly decreases circulating oxLDL concentrations and that such an effect is independent of the intensity (dose) and lipophilicity of statin. Meta-analysis of 3 clinical trials showed that statin treatment did not change serum levels of IgM and IgG antibodies to oxLDL.

The results of earlier studies suggested that elevated levels of circulating oxLDL might be associated with preclinical arterial injury, coronary and peripheral arterial atherosclerosis, and ASCVD outcomes [59]. Circulating levels of oxLDL are associated with all stages of atherosclerosis, from the earliest asymptomatic phases such as endothelial dysfunction to the clinical manifestations of ASCVD and events. It has been reported that oxLDL levels were associated with ASCVD risk factors including hyperlipidemia, hypertension, diabetes, obesity, and metabolic syndrome [60, 61].

After the first small study published in 2004 showing that the level of circulating oxLDL was significantly decreased by treatment with statins (fluvastatin and pravastatin) and that this effect was independent of their lipid-lowering effect [62], a number of mostly small studies was published supporting the same finding. In recent years, several smaller studies were performed showing the beneficial effects of statins on oxLDL [63] suggesting that high-dose atorvastatin and rosuvastatin induce similar decreases in oxLDL [64]. The pleiotropic effects of statins (e.g., antioxidative and anti-inflammatory) might have contributed to the reduction of oxLDL formation [65, 66]. For instance, since C-reactive protein (CRP) and oxLDL are interlinked in pathophysiological pathways [67], the reduction in plasma CRP levels with statins [68] could be related to the lowering of oxLDL. Furthermore, statin-induced lowering of LDLs decreases the circulating level of the substrate (i.e., LDL particles) for oxidation, and this could partially account for reduction in the generation of oxLDL.

Irrespective of cholesterol-dependent or cholesterol-independent (pleiotropic) effects of statins [69–72], plaque oxLDL levels might be associated with plaque inflammation. However, a recent study showed that plaque oxLDL levels were not associated with future ASCVD events [73]. It is important to stress that plaque levels of oxLDL were lower in patients who were treated with statins.

Based upon the results of studies showing that elevated oxLDL levels can independently predict recurrent stroke in patients with minor stroke or TIA [74], several recent studies have shown that prestroke treatment with statins can reduce serum oxLDL levels and that statins improve clinical outcomes in patients with atrial fibrillation-related acute ischemic stroke [75, 76]. Overall, the results of this meta-analysis and of previous studies may support the hypothesis that the beneficial effects of statins on ASCVD may be related, at least in part, to their ability to reduce oxLDL levels.

Antibodies to oxLDL have been associated with atherosclerosis presence, progression, and related clinical events, with the latter association being independent of and additive to LDL-C levels [10]. It is important to note that when normolipemic patients were treated with a high dose of atorvastatin, this resulted in a decrease in the levels of autoantibodies against oxLDL [57]. However, our meta-analysis could not find a significant effect of statins on antibodies against oxLDL. Although anti-oxLDL antibodies may have a pathogenic role in ASCVD, our results suggest that the beneficial effect of statins on ASCVD may be independent of the detrimental impact of anti-oxLDL antibodies.

This meta-analysis has some strengths and some limitations. Several studies and a relatively recently published meta-analysis have shown that increased levels of circulating oxLDL are associated with clinical ASCVD events [77], but no meta-analysis has so far investigated the effects of statin therapy on circulating oxLDL levels. This is the novelty of our analysis. A limitation is that not all studies uniformly measured and reported oxLDL values, thereby justifying the use of SMD as a summary statistic for the pooled effect size in this meta-analysis. Another limitation is that the meta-analysis of data on antibodies against oxLDL included only 3 studies (although with 2575 subjects), which might have introduced a bias towards a negative finding. Also, the PROSPERO protocol has not been preregistered for this review. Besides, the methods for measuring oxLDL concentrations in some studies included in this meta-analysis were different and might explain heterogeneity in our findings, although the use of standardization analysis reduces this error. Additionally, LDL oxidation can be affected by a number of concomitant factors, such as obesity, triglyceride levels, systemic inflammation, or LDL particle size, which were not fully evaluated in this study. Furthermore, dietary patterns, level of physical activity, smoking, and some drugs may modify LDL oxidation, which have not been considered in the included studies.

## 5. Conclusions

This meta-analysis suggests that patients treated with statins have significantly lower circulating concentrations of oxLDL and that this effect is not related to the intensity or lipophilicity of the statins used. Beyond well-known reduction in LDL-C, the beneficial effect of statins may partly be associated with the reduction of oxidative modifications of LDL and its effect on different stages of the atherosclerotic process. Further studies should address the association between statin-induced reduction of oxLDL and its effect on cardiovascular outcomes, particularly in patients with diabetes, metabolic syndrome, and chronic kidney disease. Furthermore, the effect of other lipid-lowering drugs, such as ezetimibe, PCSK9 inhibitors, and fibrates, on oxLDL levels also merits further investigation.

## Figures and Tables

**Figure 1:** Flow chart of studies identified and included in meta-analysis.

**Figure 2:** Quality of bias assessment of the included studies in this meta-analysis.

**Figure 3:** (a) Forest plot displaying standardized mean difference and 95% confidence intervals for the effect of statins on circulating concentrations of oxidized LDL. (b) Leave-one-out sensitivity analyses for the effect of statins on circulating concentrations of oxidized LDL.

**Figure 4:** Forest plot displaying standardized mean difference and 95% confidence intervals for the effect of statins on (a) IgM antibodies to oxidized LDL and (b) IgG antibodies to oxidized LDL.

**Figure 5:** Random-effects metaregression for assessing the effect of (a) treatment duration, (b) baseline level, and (c) delta LDL-C.

**Figure 6:** Funnel plot detailing publication bias in studies reporting the effect of statin treatment on circulating concentrations of oxidized LDL.

**Table 1:** Characteristics of studies that measured circulating concentrations of oxidized LDL and MDA LDL.

Study, year	Study design	Follow-up	Treatment	Control	Clinical outcome		Patients	No. of patients
					oxLDL	MDA-LDL		
Diepeveen et al., 2005 [31]	Double-blind randomized placebo-controlled study	12 weeks	A (40 mg/day)	Placebo	Significant decrease in serum level of oxLDL	—	Dialysis patients	23
Dogra et al., 2005 [32]	Double-blind, randomized cross-over study	6 weeks	A (40 mg/day)	Placebo	Significant decrease in serum level of oxLDL	—	T1DM with microalbuminuria	32
Dogra et al., 2007 [33]	Double-blind, randomized, placebo-controlled, parallel-group study	6 weeks	A (40 mg/day)	Placebo	Significant decrease in serum level of oxLDL	—	CKD stages 3 to 5	63
Vlachopoulos et al., 2007 [34]	Randomized, placebo-controlled, double-blind study	4 days	A (40 mg/day)	Placebo	Significant decrease in serum level of oxLDL	—	Acute systemic inflammation-induced endothelial dysfunction in hypercholesterolaemic patients	50
Singh et al., 2008 [35]	Randomized double-blind placebo-controlled study	12 weeks	A (10, 80 mg/day)	Placebo	Significant decrease in serum level of oxLDL	—	Metabolic syndrome	70
Nou et al., 2016 [36]	Randomized, placebo-controlled study	12 months	A (40 mg/day)	Placebo	Significant decrease in serum level of oxLDL	—	HIV-infected patients with subclinical coronary atherosclerosis	37
Nixon et al., 2017 [37]	Multicenter, prospective, randomized, double-blind, placebo controlled, cross-over pilot study	20 weeks	A (20 mg/day)	Placebo	Significant decrease in serum level of oxLDL	—	HIV-infected patients	146
deFilippi et al., 2018 [38]	Single-center randomized double-blind placebo-controlled study	12 months	A (40 mg/day)	Placebo	Significant decrease in serum level of oxLDL	—	HIV-infected patients	39
Yamada et al., 2007 [39]	Prospective randomized controlled study	6 months	A (10 mg/day)	Placebo	—	Significant decrease in serum level of MDA-LDL	CHF	38
Oka et al., 2008 [40]	Randomized controlled study	12 weeks	A (10 mg/day)	Only diet therapy	—	Decrease in serum level of MDA-LDL	CAD and hyperlipidemia	48
El-Sisi et al., 2015 [41]	Single-center, blind randomized investigational study	3 months	A (20 mg/day)	Conventional therapy of HF	Significant decrease in serum level of oxLDL	—	CHF	48
Andreou et al., 2010 [42]	Randomized placebo-controlled study	1 month	R (10 mg/day)	Placebo	Significant decrease in serum level of oxLDL	—	CHF	39
Erbs et al., 2011 [43]	Randomized, double-blind, and placebo-controlled study	12 weeks	R (40 mg/day)	Placebo	Significant decrease in serum level of oxLDL	—	CHF	40
ter Avest et al., 2005 [44]	Double-blind, randomized cross-over study	12 weeks	R (40 mg/day)	Placebo	Significant decrease in serum level of oxLDL	—	Familial combined hyperlipidemia	36
Hileman et al., 2016 [45]	Randomized, placebo-controlled trial	48 weeks	R (10 mg/day)	Placebo	Increase in serum level of oxLDL	—	HIV-infected patients	147
Abe et al., 2011 [46]	Randomized, prospective, open-label, parallel-group, controlled study	6 months	R (10 mg/day)	Patients without statin prescription	—	Significant decrease in serum level of MDA-LDL	Diabetic nephropathy	101
Rydén et al., 2012 [47]	Randomized, double-blind, placebo-controlled study	6 weeks	S (40 mg/day)	Placebo	Significant decrease in serum level of oxLDL	—	Mild to moderate hypercholesterolemia	76
Krysiak et al., 2011 [48]	Prospective, randomized, placebo-controlled study	90 days	S (40 mg/day)	Placebo	Significant decrease in serum level of oxLDL	—	Isolated primary hypercholesterolemia	49
Kirmizis et al., 2010 [49]	Prospective, controlled, single-center study	6 months	S (10 mg/day)	Patients without prescriptions	Significant decrease in serum level of oxLDL	—	Patients with chronic hemodialysis	50
Kishimoto et al., 2010 [50]	Randomized controlled study	16 weeks	S (5, 10 mg/day)	Patients without prescriptions	Significant decrease in serum level of oxLDL	—	Patients with chronic hemodialysis	37
Ichihara et al., 2002 [51]	Randomized, double-blind, placebo-controlled study	6 months	F (20 mg/day)	Placebo	—	Significant decrease in serum level of MDA-LDL	T2DM hemodialysis patients with normal serum lipid levels	22
Yoshida et al., 2010 [52]	Randomized controlled study	4 weeks	Pi (2 mg/day)	Patients without prescriptions	—	Significant decrease in serum level of MDA-LDL	Chronic smokers	30
Janatuinen et al., 2004 [53]	Randomized, double-blind, placebo-controlled study	4 months	P (40 mg/day)	Placebo	Significant decrease in serum level of oxLDL	—	T1DM	42
Tani et al., 2005 [54]	Prospective, single-center, randomized, open study	6 months	P (5-20 mg/day)	Patients without prescriptions	—	Significant decrease in serum level of MDA-LDL	Stable coronary artery disease	75
Ky et al., 2008 [55]	Randomized, parallel-arm, double-blind, placebo-controlled study	16 weeks	P (40 mg/day); A (10, 80 mg/day)	Placebo	Significant decrease in serum level of oxLDL	—	Hypercholesterolemic patients	106

Abbreviation: A: atorvastatin; OxLDL: oxidized low-density lipoprotein; MDA-LDL: malondialdehyde-modified low-density lipoprotein; T1DM: type 1 diabetes mellitus; CKD: chronic kidney disease; HIV: human immunodeficiency virus; CHF: chronic heart failure; CAD: coronary artery disease; HF: heart failure; R: rosuvastatin; CHF: chronic heart failure; S: simvastatin; T2DM: type 2 diabetes mellitus; F: fluvastatin; Pi: pitavastatin; P: pravastatin.

**Table 2:** Characteristics of studies that measured antibodies to oxidized LDL and MDA LDL.

Study, year	Study design	Follow-up	Treatment	Control	Clinical outcome		Patients	No. of patients
					AuAb-oxLDL	AuAb-MDA-LDL		
Tsimikas et al., 2004 [56]	Randomized, double-blinded, placebo-controlled study	16 weeks	A (80 mg/day)	Placebo	—	Significant increase in serum level of AuAb-MDA-LDL	ACS	2341
Kuklinska et al., 2010 [57]	Randomized prospective open-label study	3 months	A (80 mg/day)	Statin free patients	Serum level of AuAb-oxLDL decreased, but the alterations were not significant	—	Normolipidemic patients	56
Rodenburg et al., 2006 [58]	Double-blind, randomized placebo-controlled study	2 years	P (20-40 mg/day)	Placebo	—	Significant changes in serum level of AuAb-MDA-LDL	Children with familial hypercholesterolemia	178

Abbreviation: A: atorvastatin; AuAb-oxLDL: autoantibodies against oxidized LDL; AuAb-MDA-LDL: autoantibodies against malondialdehyde-modified LDL; NICM: nonischemic cardiomyopathy; ACS: acute coronary syndrome; P: pravastatin.

**Table 3:** Subgroup analysis based on treatment duration, statin type, lipophilicity, and intensity.

Subgroup		SMD	95% CI	*p* value	*I* ^2^ value (%)
Statin type	Atorvastatin	-1.85	-2.36, -1.33	<0.001	86.86
	Simvastatin	-4.52	-6.69, -2.35	<0.001	95.92
	Rosuvastatin	-1.36	-2.36, -0.372	0.007	93.90
	Fluvastatin	-3.19	-4.46, -1.93	<0.001	0
	Pitavastatin	-2.90	-3.93, -1.87	<0.001	0
	Pravastatin	-2.10	-3.96, -0.253	0.026	94.58
Statin lipophilicity	Hydrophilic	-1.57	-2.37, -0.77	<0.001	93.23
	Lipophilic	-2.37	-2.91, -2.83	<0.001	90.38
Statin dose	High	-1.95	-2.58, -1.33	<0.001	84.27
	Low to moderate	-2.25	-2.85, -1.66	<0.001	93.42
Treatment duration	>12 months	-1.73	-2.23, -1.24	<0.001	84.75
	<12 months	-2.67	-3.41, -1.93	<0.001	94.32

## Data Availability

There is no primary dataset associated with this study.

## Supplementary Materials

Supplementary Materials Table S1: summary of the search strategy. Table S2: summary of the strength of evidence using the Grade of Recommendations, Assessment, Development and Evaluation (GRADE) system.
